The article "Event-Related Potential Sensing Analysis on the Risk Perception and Decision-Making by Grassroots Managers in Different Fatigue States" was published in 2021. Journal: J Healthc Eng.

# Event-Related Potential Sensing Analysis on the Risk Perception and Decision-Making by Grassroots Managers in Different Fatigue States

**DOI:** 10.1155/2021/2858536

**Published:** 2021-09-23

**Authors:** Yixin Huang, Hongxia Li, Yanling Yang, Jin Wang, Janis Jansz

**Affiliations:** ^1^School of Economics and Management, Yan'an University, Yan'an 716000, China; ^2^Soft Science Research Base for Green and Low Carbon Development of Energy Industry in Shaanxi Province, Yan'an University, Yan'an 716000, China; ^3^Graduate School, Xi'an University of Science and Technology, Xi'an 710054, China; ^4^Medical School, Yan'an University, Yan'an 716000, China; ^5^School of Mines: Minerals, Energy and Chemical Engineering, Faculty of Science and Engineering, Curtin University, Perth 6945, Australia

## Abstract

The risk perception and decision-making ability of grassroots managers is the key to the normal operation of enterprises. This study used event-related potential indicators (ERPs) to reveal the process of risk perception and decision-making behaviour of coal mine grassroots managers in different fatigue states. The ERP components, such as CNV, P300, MMN, and FRN, during risk perception, decision-making, and postperception periods were obtained and evaluated. The peak value and variation characteristics of ERP components of grassroots managers under fatigue and nonfatigue conditions were analysed. Accordingly, the effectiveness of decision-making behaviour in different periods was determined. The results showed that the P300 component is a key indicator in measurements of the deviation of grassroots managers' decision-making behaviour, and FRN could reflect the negative emotions in the decision-making process and reflect the sensitivity of the risk perception of grassroots managers. There was a significant difference between the peak voltages of the ERP components of the grassroots managers in fatigue and nonfatigue states. The peak voltage of the ERP components of the grassroots managers in a fatigue state was generally greater than 10 *μ*V; therefore, the quality of decision-making by the grassroots managers could be evaluated according to the characteristics of the ERP components. This study provides a risk decision-making reference for grassroots managers of coal mine enterprises.

## 1. Introduction

In recent years, infrastructure construction in developing countries has been in full swing. A large number of large geotechnical engineering projects in the fields of water conservancy, mining, and underground engineering are under construction [1–4]. In this context, the contradiction between the construction needs of geotechnical engineering and the relatively insufficient technology or lagging management of engineering in developing countries has become prominent [5]. This contradiction leads to frequent accidents in the process of engineering construction in developing countries. Taking China as an example, engineering accidents in China has been highly detrimental in recent years, resulting in high economic losses and casualties. Of these, the proportion of accidents involving geotechnical engineering has been as high as over 10% [6]. Among these engineering accidents, coal mine accidents in China have always been the focus of society as a whole [7]. According to statistics in the first half of 2020, in Shanxi Province alone, there were 5 coal mines with fatal accidents with 8 deaths, and 150 mines were suspended for rectification. Ensuring the safety of coal mine workers is the key to ensuring the healthy and sustainable development of mining enterprises.

Risk decision-making analysis is a key link in enterprise quality management and operational risk assessment [8, 9]. To perform risk analysis and decision-making processes, a multiattribute analysis method must be established, and the most important influencing factors affecting enterprise operational risks must be screened out [10, 11]. Xiong et al. analysed the causes of 50 typical engineering accidents and found that 55.6% of the accidents were caused by human factors [6]. Long-term monotonous labour and harsh environments can easily lead to heavy mental stress and physical or mental fatigue in miners [12, 13]. For some grassroots managers, long-term fatigue could cause them to have a negative and insensitive attitude to coping with work. Therefore, some grassroots managers could lose the sensitivity of risk perception in daily work, and they would exhibit incorrect behaviours when coping with risk decisions. This would directly cause production accidents [14]. As a result, poor decision-making behaviours would occur when dealing with risks, which would directly cause accidents. Hence, grassroots managers' perception of risks and their ability to make correct decisions are important factors in the prevention of safety accidents. An increasing number of research institutes of coal enterprises are committed to integrating the physiological response of managers under specific risk stimulus conditions with the evaluation system of decision-making and to studying the physiological components and change indicators of managers in the process of risk decision-making [15]. Accordingly, the work status and behaviour of managers are identified, and the decision-making behaviours of managers are scientifically evaluated.

It is beneficial to use modern experimental research techniques, such as event-related potentials (ERPs) [16], magnetoencephalograms [17], and functional magnetic resonance imaging [18], to analyse the physiological indicators of the decision-making process of human beings. Among these technical methods, ERP research has penetrated many fields, such as psychology, physiology, medicine, neuroscience, and artificial intelligence and is increasingly recognized by people [19–21]. As early as the 1970s, Squires et al. proposed the concept of ERPs, which recorded brain evoked potentials from the surface of the skull using averaging and superposition technology to reflect the neuroelectrophysiological changes in the brain during the cognitive process [22]. Given the close relationship between ERPs and the cognitive process, ERPs are considered to be windows into the mental activities of people. With the continuous application of ERP experimental research, an increasing number of ERP components have been discovered. Walter et al. first proposed the contingent negative variation (CNV) component during the ERP testing process in 1964 [23]. In addition to the CNV component, components such as MMN, P300, and FRN are also widely used in ERP tests [24–27]. In recent decades, an increasing number of people have applied ERP methods to the field of engineering safety management. These studies mainly focused on the unsafe behaviour of subjects and the identification of risk patterns of physiological indicators. For instance, ERP tests are used to evaluate the physiological indicators of the driver in each stage of “cognition-perception-response” [28]. ERP experimental research in the field of coal mine safety management mainly focuses on the safety psychology and unsafe behaviour of miners, discussing the influence of the safety psychological capital of miners on unsafe behaviour from the perspective of brain nerve mechanisms [29].

Although some research progress has been made in engineering safety analysis by ERP technology, there are still few studies on risk perception and decision-making with grassroots managers as the subjects. Especially in coal mining engineering, various coal mine dynamic disasters, such as coal bumps [30] and gas outbursts [31] seriously threaten the personal safety of workers. Therefore, it is of great significance to evaluate the risk perception and decision-making process of coal mine grassroots managers. In this study, several grassroots managers of a coal mine are selected as subjects, and some representative risk decision-making cases in daily work are selected as stimulus conditions. The ERP tests of risk decision-making under fatigue and nonfatigue states of grassroots managers are carried out in groups. The experimental process is divided into the risk perception period, decision period, and postperception period. The characteristics of ERP components, such as CNV, P300, MMN, and FRN, of the participants of the three periods are studied, and the peak voltage and change rule of different ERP components are statistically analysed. Accordingly, ERP component index thresholds that can evaluate the risk decision-making behaviour of grassroots managers in coal mines are proposed. This study provides a reference for the risk decision-making of grassroots managers of coal mine enterprises.

## 2. Experimental Design and Data Processing

### 2.1. Experimental Design and Preparation

Due to the complexity of mining work, grassroots managers in coal mines have a low sense of risk perception and a high rate of decision errors. The decision-making level of grassroots managers is directly related to the safety of miners and the production efficiency of coal mines. Evaluating the risk perception and decision-making level of grassroots managers is important to ensure the safe and efficient production of coal mines.

ERPs are special brain evoked potentials that use the potential of the brain caused by multiple or diverse stimuli by deliberately giving stimuli a special psychological meaning. It reflects the changes in the neurophysiology of the brain during the cognitive process. It is also called cognitive potential, which refers to the brain potential recorded from the surface of the head when people perform cognitive processing on a certain subject. ERP experiments are conducted to clarify the risk perception and decision-making level of grassroots managers in coal mines during the decision-making process. Grassroots managers such as trade union chairmen, mining team captains, and ventilating team captains of multiple coal mines are selected as the subjects. The ERP experimental system of the risk perception and decision-making of coal mine managers is constructed as follows: the ERP test machine (Version: B-Alert 3.0) is connected in parallel with the sensor electrodes, and the terminals are connected to the computer. The E-Prime 2.0 program platform is used to collect and analyse ERP signals, and the cases matching the complex coal mine project decision events are selected as the stimulus conditions. The ERP experiment test system for risk perception and decision-making is shown in Figure 1, and the ERP experiment equipment, material library, and stimulus conditions required for the specific decision and perception process are shown in Figure 2.

This experimental study is divided into ERPs testing of risk perception and risk decision-making. The characteristics of ERP signal components were analysed during risk perception and decision-making. This experiment was divided into risk perception and risk decision-making ERP testing and analysed the characteristics of ERP signal components in the early stage of risk perception and the risk decision-making process. The design experiment was divided into two groups: the risk decision ERP test group and the risk perception ERP test group. The risk perception ERP experiment was based on the completion of the risk decision experiment. The decision-making ERP experiment was divided into 9 control groups, and 12 grassroots managers with experience in large-scale coal mine project construction were selected. The stimulation conditions were divided into positive and negative groups (control group), with 6 subjects in each group. The test results are divided into three categories: “correct,” “positive meaning shift,” and “negative meaning shift.” Take the ERPs experiment in the process of risk decision-making under fatigue stimulus conditions as an example. Twelve subjects in each group will be divided into groups to carry out “positive” and “negative” stimulus experiments; that is, the subjects will make decisions during the exhausted state and the good state to test fatigue. Auditory response and visual induction response under loading conditions such as stress, simultaneous handling of multiple events, and crisis attributes comprehensively evaluate the risk decision-making and perception level of coal mine managers in the risk decision-making process.

The ERP signals were analysed through the E-prime 2.0 program platform. The important nodes and fluctuation characteristics of the signal data are marked. According to the decision-making process, the experiment is divided into three stages: consciousness period (Block 1), decision period (Block 2), and postperception period (Block 3). To exclude the influence of time factors on risk perception and changes in ERP composition characteristics, the experiment time was limited to 60 s. The duration of the consciousness period (Block 1), decision period (Block 2), and postperception period (Block 3) were 20 s, 30 s, and 10 s, respectively. To ensure the correlation between the two experiments and the validity of the data of the subjects, the test subjects rested for 5 minutes after the first experiment. To ensure the relevance of the two experiments and the validity of the test data, the rest period between groups was set to 5 minutes. During the experiment, key nodes and abnormal signal zones are manually selected, and different types of ERP data are recorded at different times. This is helpful for the follow-up observation of the ERP component characteristics of grassroots managers during the risk perception stage and decision-making stage.

### 2.2. ERP Signal Filtering and Analysis Method

When the brain performs tasks or receives external stimuli, it generates electrical signals (usually 1.0 to 100 mV). By arranging potential sensors on different parts of the brain surface, the weak electrical signals can be filtered and amplified, and a continuous waveform can be obtained. These electrical signals could be divided into electroencephalograms (EEGs) and event-related potentials (ERPs). EEG scans show the continuous brain electrical signal waveform obtained by the electrode sensor, while ERPs depict the electrical signal waveform of the evoked potentials before and after the trigger event. This paper carried out an ERP experiment on the risk decisions and perceptions of grassroots managers in fatigue and nonfatigue states. Waveforms of ERP components, such as contingent negative variation (CNV), P300, mismatch negativity (MMN), and feedback-related negativity (FRN), are obtained during the risk decision-making process of grassroots managers in coal mines. The peak voltage of different components of coal mine grassroots managers during the decision-making process was extracted. The level of risk perception and decision-making quality of coal mine grassroots managers are judged. This provides support for the construction of an intelligent risk management and control system for complex coal mine projects.  Figure 3 shows the experimental methods of ERPs and waveforms of ERP signals.

During the ERP test of coal mine grassroots managers, the frequency of ERP components fluctuated frequently due to the stimulation of external conditions and events. ERP components are different under loading conditions, such as fatigue, stress, multievent handling, aural induction, and visual induction. In coal mine production, the decision-making events of grassroots managers include the replacement and maintenance dates of common equipment, turn-off dates of miners, safety qualification checks for miner positions, and daily workload arrangements. Different decision events correspond to different test potentials, so the ERP tests are performed on the subjects using the one-by-one measurement method. The extracted signal components mainly include CNV, MMN, and P300. In addition, the N4 component (related to semantic understanding matching), N2 component (related to auditory induction), and FRN component (related to intention processing) are observed. Published ERP research shows that the early CNV component mainly determines the concentration and response level of the subject in the early stage of decision-making. N2 reflects the early visual image of decision-making by the subject. MMN reflects the auditory image in the decision-making process of the subject. P300 reflects the concentration and response level during the decision period. The late CNV component can measure the level of alertness of the subject. This paper mainly analyses the characteristics of ERP signals in the risk perception and decision-making process of coal mine grassroots managers. The ERP components in the awareness period (Block 1), decision period (Block 2), and postperception period (Block 3) during the experiment are compared. The feature of voltage change reveals the risk perception and decision-making of coal mine grassroots managers to reveal the risk perception and decision-making rules of coal mine grassroots managers.

## 3. ERP Characteristics of Decision-Making by Grassroots Managers

### 3.1. Peak Voltage Variations of CNV and MMN during the Risk Perception Period

To explore the influence of negative stimuli on the risk decision-making of grassroots managers in coal mines, the experimental grassroots managers were divided into two groups: a nonfatigue group and a fatigue group. The following takes equipment replacement as a decision event as an example to explain the test process. First, a predictive signal *S*1 (conditional stimulus) is applied to the subject before providing a decision-making event; then, the command signal *S*2 is applied when the decision-making event is executed. The two stimuli are separated by 1 to 2 seconds. The recorder will obtain ERP signals, such as CNVs and MMNs, during the process. In the tests, subjects numbered *P*1 to *P*6 belong to the nonfatigue group, and subjects *P*7 to *P*12 belong to the fatigue group. The test process is divided into three periods: Block 1 (risk perception period, 0–220 s), Block 2 (decision-making period, 20–550 s), and Block 3 (postperception period 50–660 s). The changes in CNV and MMN were analysed during the risk perception period and the results are provided below.

The CNV change characteristics and peak voltage results of the grassroots managers during the risk perception period (Block 1) are shown in Figure 4. The 6 subjects in the nonfatigue group all produced CNV components. The peak voltage time ranges 9.15∼11.23 s, and the peak value ranges 6.5∼10.1 *μ*V. For the fatigue group, only 4 subjects produced CNV components, the peak time ranged from 11.26 to 11.86 s, and the peak value ranged 5.5 *μ*V∼5.9 *μ*V. Taking Subject 5 in the nonfatigue group and Subject 10 in the fatigue group as examples, the impact of fatigue on the decision-making behaviour of grassroots managers in the coal mine is analysed. During the risk perception period, the CNV component induction time of Subject 5 is 11230 ms with a duration of 50 ms, and the peak value reaches 10.1 *μ*V with an amplitude of 12.1 *μ*V. CNV gradually stabilized after the peak. The changing trend of CNV of Subject 10 is consistent with that of Subject 5. However, the CNV component induction time is 11260 ms with a duration of 50 ms, and the peak value is 5.8 *μ*V with an amplitude of 7.7 *μ*V. The CNV component of Subject 10 induces a longer latency period and lower peak voltage, which indicates that the negative wave of the CNV component is more active in the nonfatigue condition during the risk perception period (Block 1). Therefore, the characteristics of the CNV component can be used to judge whether the grassroots managers in coal mines are in a state of fatigue during the risk perception period. During the construction of risk management and intelligent control systems for coal mines, it is possible to consider designing and installing matching potential sensors in miners' helmets to monitor the characteristics of the CNV components in real-time and establish scientific risk management and early warning platforms based on this.

The MMN component is related to the early preprocessing activities of auditory information, reflecting the activation process of the primary auditory cortex and adjacent superior temporal gyrus. The peak MMN component results of 6 nonfatigue subjects during the risk perception period are shown in Figure 5. In the tests, the subjects in the fatigue group produced no MMN components during the perception period, while 4 subjects in the nonfatigue group produced MMN components (the peak voltage was negative). This indicates that the nonfatigue group has significantly stronger anti-interference ability than the fatigue group in terms of auditory evoked potential during the tests. Therefore, it can be considered to judge the working status of grassroots managers in coal mines during the risk perception period with the characteristics of MMN components.

### 3.2. Peak Voltage Variations of P300 and FRN during the Decision-Making Period

It is of great significance to study the characteristics of ERP components in the process of risk decision-making of grassroots managers in coal mines. The P300 component was discovered and proposed by Sutton et al. in 1965 and belongs to the third positive wave. P300 usually appears approximately 300 ms. Generally, P300 is widely used in the judgement, early diagnosis, and adjuvant treatment of various diseases caused by brain injury. At present, most studies focus on the use of P300 to study dementia diseases. Therefore, the P300 component characteristics in the decision-making period of grassroots managers in coal mines are the key information indicators for judging the biased stimulus of decision-making behaviour. (Figure 6(a)) shows the characteristics of the P300 component during the decision-making period of the subjects, and the statistical analysis of the peak voltage of the P300 component during the decision-making period of 12 subjects is shown in (Figure 6(b)). The results show that the P300 component induction levels of the 6 subjects in the nonfatigue group are relatively consistent, with an average induction time of 300.16 ms and a peak value of 8.491 *μ*V. The P300 component induction level of the 6 subjects in the fatigue group was different. The earliest and latest induction times are 300 and 300.45 ms, respectively. The average induction time was 300.22 ms, and the average peak voltage was 13.19 *μ*V. Therefore, the P300 component of the test subject has relatively high voltage feedback in the fatigue state, which indicates that the fatigue test subject has weak anti-interference ability, insufficient concentration, and weak decision-making willingness. The feedback of coal mine managers in the state of fatigue to emotional motivation is more obvious. In the construction of the coal mine risk management and intelligent perception system platform, the peak voltage of the measured P300 component can be considered as the threshold to determine whether the risk decision of coal mine grassroots managers under fatigue and nonfatigue is effective.

The FRN component is the feedback negative wave in the midline area of the forehead of the scalp. The negative wave component appears within approximately 200–400 ms after the feedback stimulus is presented. FRN reflects the difference between expected and actual results. It can represent a negative wave component induced by negative feedback stimuli such as behaviour errors. Gehring et al., 2002, proposed the emotional motivation hypothesis that FRN reflects the evaluation process of the meaning of emotional motivation. Therefore, FRN can reflect the negative emotions of coal mine managers when they make the wrong risk decisions in this study.  Figure 7 shows the FRN component signal characteristics and peak voltage comparisons of 12 subjects in the risk decision period. The results show that subject P4 in the nonfatigue group fails to induce FRN components. The FRN component induction time of the remaining five subjects in the nonfatigue group was concentrated at 312 ms, with an average peak voltage of -6.34 *μ*V. Six subjects in the fatigue group all induced FRN components, and the induction time was 320 ms after stimulation with an average peak voltage of −2.67 *μ*V. In the fatigue state, the FRN component induction time of subjects was relatively late. The above research shows that, during the decision-making period of the nonfatigue group, the subjects were more focused and motivated to make decisions, and they were less willing to make gambling decisions. These fatigued subjects have inattention, weak decision-making motivation, and strong decision-making behaviour and have strong negative feedback on incorrect decision-making behaviour. Therefore, the FRN component can be considered the risk feedback signal of the wrong decision in the risk management and intelligent perception system of complex projects in coal mines. According to the test results, the peak value of the FRN component voltage of coal mine managers during the risk decision period can be used as the critical value. This can verify the negative sentiment of the wrong decision-making behaviour of decision-makers.

### 3.3. Peak Voltage Variations of CNV and P300 during the Postperception Period

The feedback period after risk decision-making is the postperception process of decision-making behaviour. The periods of 50∼60 s and 110∼120 s in the experiment were the postperception period of the nonfatigue group participants and the postperception period of the fatigue group participants. The process is the process of thinking and feedback on risk decision awareness in the early stage of decision-making, and it is also the process of rethinking to improve cognitive risk perception ability. Therefore, in this experiment, the CNV component and the P300 component of the primary management subjects were the main analysis targets. During the postsensing period, the peak voltage and change process of the primary coal mine managers' components are shown in Figures 8 and 9. In the test results of the nonfatigue group, 5 subjects induced CNV components in the late stage, and the voltage peak was at 11.05–12.43 *μ*V. The CNV induction time of 6 subjects in the fatigue group was generally later than that in the nonfatigue group. The CNV component of the nonfatigue group participants in the postrisk perception period had the characteristics of short latency and high potential peak, indicating the decision-making efficiency of the managers in the nonfatigue group was high during the decision recall process; also, the ERPs information response was relatively rapid, while the fatigue group ERPs information response was delayed and managers exhibited a lack of concentration.

The P300 component characteristics in the postperception period are the process of rethinking the decision-making behaviour deviation stimulus.  Figure 9 shows the P300 component characteristics of the 12 subjects in the postperception period. Two subjects in the nonfatigue group did not induce the P300 component (peak voltage is 0), and the remaining 4 subjects all obtained the P300 component and average peak voltage in approximately 277 ms. The P300 component of the fatigue group was later than that of the nonfatigue group, which shows that the grassroots coal mine managers significantly stimulated the decision-making behaviour deviation under the fatigue state.

## 4. Conclusions

ERP tests on the risk perception and decision-making behaviour of grassroots managers in coal mines were conducted in this paper. The characteristics of ERP components, such as CNV, P300, MMN, and FRN, of the participants were studied in three periods; also, the peak voltage and pattern of change in different ERP components were statistically analysed. The main conclusions are described below.

1. The risk decision-making process of coal mine grassroots managers can be divided into perception periods, decision-making periods, and postperception periods according to the characteristics of ERP information. CNV and MMN components in the perception period can reflect the sensitivity of the decision-making subject's risk perception. P300 and FRN components in the decision period can reflect the auditory induction, anti-interference ability, and negative emotional feedback of the decision-making process. The CNV and P300 component characteristics in the postperception period can verify the decision-making behaviour deviation through the state of physiological indicators.
2. There is a significant difference in the peak voltage of the risk decision ERPs of coal mine managers under fatigue and nonfatigue states. The results show that the P300 component is a key information indicator reflecting the deviation stimulus of decision-making behaviour during the decision-making period. The peak voltage of the P300 component under the fatigue state is generally greater than 10 *μ*V. The peak value of the FRN component voltage in the fatigue state is generally less than −6.0 *μ*V. Therefore, the P300 component and FRN component of the grassroots managers can be set as the respective thresholds to determine whether the decision-making behaviour is reasonable and effective.
3. The CNV component and P300 component in the postperception period reflect the manager's process of rethinking the deviation in risk perception and decision-making behaviour. Therefore, the corresponding threshold can be set in the coal mine enterprise risk management and intelligent decision-making system platform. After the person completes the decision-making behaviour, the person's fatigue state can be judged by the induction time of these two ERP components, and the deviation in decision-making deviation can be verified.

## Figures and Tables

**Figure 1:** ERP experimental equipment and simulated stimulation conditions.

**Figure 2:** Experimental stimulation conditions and risk decision process.

**Figure 3:** Experimental methods of ERPs and waveforms of ERP signals.

**Figure 4:** Changing characteristics and peak voltages of the CNV components of grassroots managers in coal mines during the risk perception period.

**Figure 5:** Changing characteristics and peak voltages of the MMN component of grassroots managers in coal mines during the risk perception period.

**Figure 6:** P300 component characteristics and peak voltage comparison of coal mine grassroots managers during the risk decision period.

**Figure 7:** FRN component signal characteristics and peak voltage comparison of coal mine grassroots managers during the risk decision period.

**Figure 8:** Comparison of CNV component signal characteristics and peak voltages of coal mine managers in the postsensing period.

**Figure 9:** P300 component signal characteristics and peak voltage comparison of coal mine grassroots managers in the postperception period.

## Data Availability

The data that support the findings of this study are available from the corresponding author upon reasonable request.
